# Research on B2C Online Marketing Mode based on Multimodel Fusion and Intelligent Big Data Analysis Method

**DOI:** 10.1155/2022/8868722

**Published:** 2022-07-30

**Authors:** Jianhua Wei

**Affiliations:** School of Management Engineering and Business, Hebei University of Engineering, Handan, Hebei, China

## Abstract

B2C online marketing mode is the development trend of future marketing. The key to improve the efficiency of such a mode is to make efficient use of the current large-scale data and mining the corresponding potential value. To control the cost of B2C online marketing mode, this paper analyzes the UJRP model and proposes a hybrid bat difference algorithm (BADE). Experimental results are verified the effectiveness of the proposed method in diversity and cost control. Furthermore, we utilize multimodel fusion strategy (linear weighted fusion) to achieve better performances in B2C online marketing on cost than BADE method. Finally, in the random and diverse online marketing environment, such an improved method can provide the decision-makers of B2C online marketing mode with more flexible choices.

## 1. Introduction

At present, there are generally two channels for the formation of an online marketing mode. One is the offline traditional marketing mode (such as physical stores), and the other is directly born on the Internet platform (such as Amazon and Tmall). No matter which channel forms the online marketing model, its business model is inseparable from Internet e-commerce B2B and B2C. E-commerce originated in Europe and America. In the initial stage, the B2C online marketing mode is difficult due to the lack of resources and relevant technical knowledge. Fundamentally speaking, people's understanding of it in this period is only a supplement to the traditional offline marketing model and only exists as an offline subsidiary. The online marketing model is still in a period of fragmentation and accumulation and has not yet formed a scale effect.

Compared with B2B (business to business), which relies on the exchange of products and information between enterprises through the Internet, B2C (business to customer) has unique advantages for the terminal retail link of industry and commerce. B2C is what we often call the online commercial retail model of selling products directly to consumers [1]. For example, in China, through traditional B2C websites such as Tmall, customers can not only make online orders and appointments through the network but also realize the order binding, online payment, and other consumption behaviors of the third-party trading platform. With the increasing number of data, B2C has increasingly become an important branch to promote the development of the world's e-commerce industry and has brought new opportunities to all walks of life, especially the development and transformation of the traditional manufacturing industry [2].

B2C online marketing mode should be said to be a new business form born under the continuous penetration and drive of Internet technology after the development of traditional industrial and commercial industries to a certain period. Although it is an emerging model, it still has its inherent shortcomings. The operation and development of the B2C online marketing mode is always inseparable from the traditional marketing mode and the offline resources of suppliers [3]. Today, with the rapid development of all walks of life, how to make up for their own shortcomings is the focus of future development.

The joint replenishment problem on e-commerce with operational efficiency loss is an extended research based on the joint replenishment problem (JRP), which applies the joint replenishment problem with uncertain demands (UJRP) to the B2C online retail industry, The purpose is to coordinate the purchase frequency of different commodities by grouping, so as to better realize the coordinated operation of “purchase, storage, and sales” of online retailers, so as to effectively reduce the total cost of system operation [4].

Therefore, combined with the operation practice of B2C online marketing mode, this paper puts forward an integrated optimization model of multiproduct procurement operation considering the operation efficiency and loss as the starting point, which integrates and optimizes the core links of the three supply chains of collection, storage and sales, so as to effectively reduce the overall operation cost of the system and realize an efficient and accurate B2C online marketing mode combined with big data analysis. Under the background of “Internet +” and big data, from the perspective of data analysis, explore the construction of an efficient utilization system of B2C online marketing mode, with a view to promoting the quality of offline marketing mode in the information environment, enriching the practice of B2C online marketing mode, and accelerating the informatization process of this emerging mode.

## 2. Related Work

The core content of the B2C online marketing mode is how to efficiently use the massive data generated online. With the improvement of the industry ecological chain and the intensification of industry competition, in order to improve the service level and reduce the loss of platform operation efficiency, the strategy of multicommodity joint procurement and operation is widely used in the B2C e-commerce industry. More scholars have also extended JRP to the field of coordinated operation of the supply chain, focusing on the coordination and optimization of the overall production operation of the supply chain with inventory control as the core [5]. Literature [6] studies the joint procurement strategy under the three-level supply chain. It can be seen that JRP gradually expands to the vertical integration and optimization of the supply chain by combining more realistic assumptions and integrating the upstream and downstream operations of the supply chain [7]. However, relevant research still focuses on traditional manufacturing industries. In recent years, the deep adjustment of global economic patterns has promoted the optimization and upgrading of industrial structure in various countries. Many scholars have also begun to pay attention to the application of JRP in more industries [8]. Cui et al. [9] proposed an integrated optimization model combining multiproduct procurement and distribution for the supply chain structure of one distribution center with multiple retailers, which has strong practical guiding significance in the fast-moving industry; in the agricultural and sideline and pharmaceutical sales industries, the quality and quantity of products are easy to change with the promotion of the purchase and marketing process. Qin et al. [10] studied the multiproduct joint pricing and inventory control when the quality and quantity of fresh agricultural and sideline products decline at the same time over time. However, at present, there are few JRP studies based on B2C e-commerce. The existing relevant studies mostly assume that the third-party platform is a free service provider, ignoring the important impact of the platform on the actual operation of online retailers [11].

Another bottleneck in the research of such problems is the design of an efficient solution algorithm [12]. JRP has been proved to be an NP hard problem [13]. In solving the model, heuristic and metaheuristic algorithms [14, 15] are mainly used, such as the Rand method [16], power, and genetic algorithm (GA) [17]. For some problems requiring exact solutions, heuristic algorithms have advantages in optimization speed and accuracy of solutions [18], but for JRP, some metaheuristic algorithms have more advantages [19]. Wang et al. used a differential evolution (DE) algorithm to solve the JRP model of fuzzy structure [17]. The algorithm shows good robustness and efficiency in solving the JRP model. However, with the increase of the problem scale, the accuracy and robustness of the DE algorithm are weakened. More researchers try to introduce intelligent algorithm into the solution [19]. Ba algorithm (BA) is an algorithm based on swarm intelligence. Inspired by the echolocation behavior of bats, it simulates the optimization and search process as the process of individual movement and prey search of population bats [20]. At first, the algorithm was mainly used to solve the structural design and optimization problems (in the engineering field). Due to its characteristics of simple implementation and few parameters, the algorithm is gradually applied to solve NP hard problems in other fields, such as production scheduling problem, optimal location problem, and pattern recognition problem [20], but the robustness of Ba is not expected. Therefore, this paper proposes a two-stage hybrid bat difference algorithm (BADE), which is different from some hybrid algorithms. Such a method does not destroy the inherent evolution process of the algorithm. The two algorithms are combined to carry out rough search and fine search respectively for different types of decision variables to produce a joint effect, which integrates the advantages of the two algorithms to a certain extent.

## 3. Method

The relationship between B2C online marketing mode and traditional marketing mode can be summarized in Figure 1.

The unified marketing model focuses on the offline marketing system and has the service experience and guarantee advantages of facing consumers directly, which is very important in the product supply chain. Although the online marketing model is fierce, it can not completely replace the role of traditional offline marketing stores, especially in terms of offline product supply and service experience guarantee. The online marketing model lacks this immediate and consistent ability.

The marketing of packaged and combined products of online marketing mode, such as group competition, package price, and special customization often depends on the offline marketing mode. Often, the offline traditional marketing model also has an online marketing strategy. This choice and cooperation will eventually form the viscosity of consumers to marketing products. In this closed-loop model, offline traditional marketing, online marketing, product suppliers, and consumers are indispensable components.

### 3.1. Model Cost

The classical JRP model mainly studies the multiproduct procurement decision-making scheme under the determined demand. The demand assumption is relatively simple [21, 22]. It is assumed that the annual fixed demand frequency of commodity *i* is *D*_*i*_, the basic replenishment cycle of each business is *t* and the joint replenishment frequency of commodity *i* is *k*_*i*_. The inventory cost in the purchase cycle can be expressed as *h*_*i*_, the corresponding formula is defined as follows:

(1) $$\begin{array}{c} C_{h}=\frac{1}{2}\sum_{i=1}^{n}k_{i}TD_{i}h_{i}. \end{array}$$

The corresponding ordering cost can be expressed as formula (2), which includes primary ordering cost and secondary ordering cost. Main ordering cost refers to the fixed cost generated by each order. This cost has nothing to do with the grouping of joint orders. The secondary ordering cost needs to consider the variable cost in each ordering process.

(2) $$\begin{array}{c} C_{o}=\frac{S}{T}+\sum_{i=1}^{n}\frac{s_{i}}{\left(k_{i}T\right)}. \end{array}$$

Then, the total cost of the JPR model is the sum of inventory cost and ordering cost, which can be expressed by the following formula:

(3) $$\begin{array}{c} TC\left(T,K\right)=C_{h}+C_{o}. \end{array}$$

With the help of mobile Internet technology and big data analysis, the BC2 online marketing environment is more complex and changeable, and the needs of customers are more fragmented and randomized. UJRP introduces the assumption of random demand based on JRP. Yes, this problem is closer to the needs of real life. Due to the uncertainty of actual demand, URJP adds shortage cost *C*_*s*_ to measure this uncertainty [23]. However, this problem needs to be based on certain assumptions, that is, the demand in B2C online marketing mode is independent, identically distributed, and subject to Gaussian distribution, and the maximum inventory level RI in the observation period can be expressed as follows:

(4) $$\begin{array}{c} R_{i}=D_{i}\left(k_{i}T+L_{i}\right)+z_{i}\sqrt{\delta_{i}\left(k_{i}T+L_{i}\right)}. \end{array}$$

Based on this assumption, the out of stock cost *C*_*s*_ can be expressed as follows:

(5) Cs=1kiTδikTi+Lifzi−zi1−Fzi.

Where *f*(*z*_*i*_) is the cumulative distribution function of the corresponding demand for commodity *I*, and *f*(*z*_*i*_) is the probability density function of the corresponding demand for commodity *i*. Then, the total cost of the UJRP model includes the sum of ordering cost, inventory holding cost, and shortage cost.

### 3.2. Model Design

As a population-based algorithm, the Ba algorithm is inspired by the echolocation behavior of bats, which simulates the optimization and search process as the process of individual movement and prey search of population bats. DE algorithm is a heuristic random search algorithm based on group difference, which has zero sign robustness in solving such problems. Bade algorithm combines the global optimization ability of BA and the robust characteristics of DE to form a two-stage algorithm. Firstly, BA is used for rough search to generate the corresponding fitness value of the current optimal bat location machine, and then the output value can be directly used as the initial input of the DE stage. In the next stage, DE plays an important role to update the best value [24]. Therefore, BADE method retains the advantages of BA and DE, and the effect is better than that of a single method. For the UJRP model, minimizing the total cost is our goal. When solving, the value of the objective function is the value of the fitness function. The detailed model flow chart is shown in Figure 2.

Specifically, the algorithm can be divided into the following steps:

(1) *Initialization*. The population position is initialized by means of uniform distribution, and the rough search starts after the initialization is completed.
(2) *The Bat Made a Rough Search*. Taking the initialized position as the starting position vector, the global optimization is carried out according to the strategy of formulas (6)–(8). Where equations (6)–(8) represent the frequency, speed, and position of the *i*-th bat, respectively.
  (6) $$\begin{array}{c} f_{i}=f_{\min}+\left(f_{\max}-f_{\min}\right)\beta , \end{array}$$
  (7) $$\begin{array}{c} v_{i}^{t}=v_{i}^{t-1}+\left(x_{i}^{t}-x^{*}\right)f_{i}, \end{array}$$
  (8) $$\begin{array}{c} x_{i}^{t+1}=x_{i}^{t}+v_{i}^{t}. \end{array}$$
(3) *Differential Variation*. The bat position vector set obtained in phase 1 is used as the DE population for mutation operation. The specific mutation strategy is shown in the following formula:
  (9) $$\begin{array}{c} v_{ij}\left(t+1\right)=pbest_{i,j}\left(t\right)+F\left(x_{r2,j}\left(t\right)-x_{r3,j}\left(t\right)\right), \end{array}$$
where *pbest*_*i,j*_ (*t*) is the optimal chromosome at the current time, *F* is the preset mutation operator, and *V*_*ij*_ (*t* *+* *1*) is the chromosome after mutation. The mutation strategy can ensure that the direction of gene mutation is closer to the optimal chromosome.
(4) *Cross Recombination*. Each dimension is compared according to formula (10) to construct a new chromosome.
  (10) $$\begin{array}{c} v_{ij}\left(t+1\right)=\left\{\begin{array}{cc} v_{i,j}\left(t+1\right), & \text{if rand}\left(j\right)\leq C_{r}\text{ or }j=\text{rand}\left(j\right),\\ x_{i,j}\left(t+1\right), & \text{otherwise}. \end{array}\right. \end{array}$$
(5) *Compare Options*. The selection operation is carried out according to the greedy rule, and the fitness (*x*_*i*_(*t*)) of each chromosome is calculated. If the fitness of the constructed new chromosome is less than that of the parent, the parent chromosome is replaced by the child chromosome, and the current optimal fitness *pbest* is output. If the *pbest* is less than *gbest*, the *gbest* is updated.

### 3.3. Multimodel Fusion Strategy

The linear weighted fusion strategy [25] is to weighted average the prediction results of a single model. By giving different weights to the prediction results of a single model classifier (the sum of the weights is 1), multiple single model prediction results are fused in order to obtain better results. The linear weighted fusion scheme can highlight the contribution of the single model classifier with better prediction results to ensure that the fusion strategy can better improve the final results. Specifically, for every single model, multiply its model weight by its sample probability and sum the values obtained by all single models to obtain the multimodel fusion results. In practical application, the multimodel fusion strategy is generally assigned manually according to experience and the effect of every single model, so its effect depends more on personal experience. Different weights are given to different models, and the fusion formula is defined as follows:

(11) $$\begin{array}{c} \sum {\text{weight}}_{i}*{\text{prob}}_{i}, \end{array}$$

where weight_*i*_ is the model weight and prob_*i*_ is the scheme output value.

## 4. Case Analysis

For the research on the actual B2C online marketing mode, the experimental data are set with reference to the previous research and real case data, as shown in Table 1. Based on the preliminary trial calculation of the initial parameter data, we can further determine the sample search space of the decision variables *k*_*i*_ and *z*_*i*_. Here, *k*_*i*_ represents the joint replenishment frequency of commodity I based on the purchase cycle, and *k*_*i*_ belongs to [1, 5]. Combined with the transaction characteristics of the online marketing mode, the types involved in the joint replenishment process are richer, so the frequency selection range should be wider.

For JRP and UJRP models, GA, BA, and DE are also used as comparison algorithms to solve them. The comparison results are shown in Table 2.

The results in Table 2 show that in solving the JRP model, compared with the four algorithms, DE and BADE have better robustness, but the variance of the DE algorithm is the smallest, the occurrence frequency of optimal value is the highest, and the performance is outstanding. When solving the UJRP model, the robustness of GA and BA algorithms (compared with solving the JRP model) is significantly weakened, but DE and BADE algorithms still show good stability. It is worth noting that in terms of searching from the optimal value, the GA algorithm appears premature when solving the two models, and the search performance is the worst; the BA algorithm only solves the JRP model, and the optimal value is similar to DE and BADE algorithm; For UJRP, bade algorithm is the best to solve the optimal value. It can be seen that bade algorithm has good solution potential for the UJRP model.

For the managers of the BC2 online marketing model, the uncertainty of the online marketing model is high, and the diversity of feasible solutions is very important. The above-given mainly evaluates the robustness and optimization ability of the algorithm from the perspective of the optimal cost. Next, we will further compare and analyze the diversity of the solution of the algorithm by investigating the diversity of product replenishment frequency (i.e., *k*_*i*_) in the feasible scheme. In the previous evaluation results, BADE and DE algorithms are selected for comparative analysis. Taking 6 products as an example, 20 groups of feasible schemes with the optimal cost function value within the error range in the solution process are randomly selected. Figures 3 and 4 are the comparison results of the diversity of feasible schemes of JRP and UJRP models, which are presented in the form of a scatter diagram. The more values of *k*_*i*_ can be taken, the more frequent the point fluctuations in the figure, which can reflect the diversity of schemes to a certain extent.

We only draw commodities with replenishment fluctuations, ignoring those that have not changed. Figures 3 and 4 show the fluctuation of bade algorithm and DE algorithm. Through comparison, it can be found that *k*_1_, *k*_4_, *k*_5,_ and *k*_6_ in bade scheme have more volatility, while the DE algorithm has only *k*_1_, *k*_4,_ and *k*_5_.

In Figures 5 and 6, for the UJRP model BADE algorithm, the volatility of *k*_4_ and *k*_5_ is obviously stronger than that of the DE algorithm, and the fluctuation range of *k*_4_ is larger. According to the comprehensive courseware, the diversity of BADE algorithm is obviously stronger than the DE algorithm for JRP and UJRP models. This also means that BADE method has stronger adaptability to practical problems. It can better optimize and adjust the cost of the B2C online marketing model with randomness.

In order to further improve the new capability of the model, the linear weighted fusion strategy is used to fuse the output of bade and DE methods, and the final effect is verified on UJRP models with different problem sizes. The results are shown in Table 3.

The following conclusions can be drawn from Table 3. For small scale, the difference between the optimal cost and average cost of BADE method is significantly larger than that of the linear weighted BADE method. The improved BADE method can control the cost well, make the average cost closer to the optimal cost, and show good stability. With the increase of the problem scale, the improved BADE method also has obvious advantages in variance and small fluctuation, which shows that this method still has good solution potential in the large-scale online marketing mode. However, this model fusion also brings computational complexity. The improved BADE method does not have advantages in running time. In general, the improved BADE algorithm still has obvious advantages in terms of performance and is still effective.

## 5. Conclusion

Under the B2C online marketing mode, to reduce the cost problem of B2C online marketing, in this paper we focus on the core part of online marketing and optimize the total cost of the system. Through the comparison between the JRP model and URJP model, a hybrid bat difference algorithm (BADE) is designed to solve different types of decision variables. By combining the advantages of BA and DE algorithms, such a method can achieves a good performance on cost control and fluctuation diversity. Multimodel fusion strategy is further added to the proposed model to leverage the potential of all methods. With such a strategy, we can obtain better results than BADE method on different scales of URJP problems.

## Figures and Tables

**Figure 1:** B2CRelationship between B2C online marketing model and traditional marketing model.

**Figure 2:** The framework of the model.

**Figure 3:** Value of BADE method *k*_*i*_ in 20 groups of JRP feasible schemes.

**Figure 4:** Value of DE method *k*_*i*_ in 20 groups of JRP feasible schemes.

**Figure 5:** Value of BADE method *k*_*i*_ in 20 groups of UJRP feasible schemes.

**Figure 6:** Value of DE method *k*_*i*_ in 20 groups of UJRP feasible schemes.

**Table 1:** Problem parameter data.

Commodity *i*	1	2	3	4	5	6
*D *_*i*_	10000	5000	3000	1000	600	100
*S*	200	200	200	200	200	200
*s *_*i*_	45	40	50	48	30	35
*h *_*i*_	3	1	1	1	1	1
*L *_*i*_	0.03	0.01	0.02	0.04	0.02	0.05
*P *_*i*_	20	13	9	10	15	7
*W *_*i*_	20	20	20	20	20	20

**Table 2:** Comparison of solution results.

	JRP				UJRP			
	GA	BA	DE	BADE	GA	BA	DE	BADE
Optimal cost	6717.1	5631.4	5631.4	5631.4	14168.1	11942.4	11680.6	11681.2
Frequency times	1	35	49	47	1	30	47	48
Variance	15.51	12.65	1.19	2.92	440.58	202.57	10.35	9.24
Average cost	6732.9	5663.5	5631.9	5634.5	15517.1	12230.3	11709.8	11699.3

**Table 3:** Comparison of UJRP results of different problem sizes.

Number	BADE				Linear weighting BADE			
	Optimal cost	Average cost	Var	Time (s)	Optimal cost	Average cost	Var	Time (s)
6	23984.1	26127.6	1076.3	18.6	23531.9	23753.6	159.4	26.5
10	34449.2	35787.4	554.58	17.6	34186.1	35600.3	520.1	21.1
15	62417.2	65097.6	473.9	19.1	62131.4	62138.39	414.2	22.3
24	144643.8	145829.2	826.1	27.5	143726.7	143826.7	182.9	22.1
29	155165.1	156933.7	1335.7	21.2	153252.7	153396.3	564.0	23.3

## Data Availability

The data that support the findings of this study are available from the author upon reasonable request.

## References

[1] Fan X. J., Wang J. B., Liu Y. (2019). Platform pricing structure of online retailers considering retailer participation. *Journal of Systems Management*.

[2] Shaouf A. A. A. (2020). The role of website visual design in predicting consumers’ purchase intentions: an empirical study in a B2C online environment. *International Journal of Online Marketing*.

[3] Tjiptoherijanto P. (2021). The Role of Communication Justice and Assertive Communication in B2C Marketplace Post Recovery Satisfaction. *International journal of social science and human research*.

[4] Liu M. L., Dan B., Zhang S. G. (2020). Information sharing in an E-tailing supply chain for fresh produce with freshness-keeping effort and value-added service[J]. *European Journal of Operational Research*.

[5] Kim S. L., Banerjee A., Burton J. (2008). Production and delivery policies for enhanced supply chain partnerships. *International Journal of Production Research*.

[6] Liu X., Cetinkaya S. (2006). A note on “quality improvement and setup reduction in the joint economic lot size model”. *European Journal of Operational Research*.

[7] Korpeoglu E., Sen A., Guler K. (2013). Non-cooperative joint replenishment under asymmetric information. *European Journal of Operational Research*.

[8] Glock C. H. (2012). The joint economic lot size problem: a review. *International Journal of Production Economics*.

[9] Cui L., Deng J., Wang L. (2018). Research on RFID investment decision based on improved joint procurement and distribution model. *China Management Science*.

[10] Qin Y. Y., Wang J. J., Wei C. M. (2014). Joint pricing and inventory control for fresh produce and foods with quality and physical quantity deteriorating simultaneously. *International Journal of Production Economics*.

[11] Wang K. J., Lin Y. S., Yu J. C. (2010). Optimizing inventory policy for products with time-sensitive deteriorating rates in a multi-echelon supply chain. *International Journal of Production Economics*.

[12] Zeng Y. R., Wan J. C., Lu S. X. (2019). Collaborative optimization of supplier selection and order allocation under joint replenishment strategy. *Control and Decision*.

[13] Cui L. G., Deng J., Zhang Y. J., Zhang Z., Xu M (2020). The bare-bones differential evolutionary for stochastic joint replenishment with random number of imperfect items. *Knowledge-Based Systems*.

[14] Liu S., Wang N. (2014). Joint reverse auction procurement and pricing decision-making under stochastic price-dependent demand. *Journal of Management in Engineering*.

[15] Cui L., Ren H., Deng J. (2020). A particle swarm algorithm for a novel B2C multi-item replenishment and delivery coordination model with fuzzy random demands. *Chinese Journal of Management Engineering*.

[16] Cui L., Wang L., Deng J. (2014). RFID technology investment evaluation model for the stochastic joint replenishment and delivery problem. *Expert Systems with Applications*.

[17] Sun C. (2022). Construction model of E-commerce agricultural product online marketing system based on blockchain and improved genetic algorithm. *Security and Communication Networks*.

[18] Vanvuchelen N., Gijsbrechts J., Boute R. (2020). Use of proximal policy optimization for the joint replenishment problem. *Computers in Industry*.

[19] Yao M. J., Lin J. Y., Lin Y. L. (2020). An integrated algorithm for solving multi-customer joint replenishment problem with districting consideration. *Transportation Research Part E Logistics and Transportation Review*.

[20] Yildizdan G., Baykan M. K. (2020). A novel modified bat algorithm hybridizing by differential evolution algorithm. *Expert Systems with Applications*.

[21] Li L., Zhang J. (2021). Research and analysis of an enterprise E-commerce marketing system under the big data environment. *Journal of Organizational and End User Computing*.

[22] Xu Z., Zhu G., Metawa N., Zhou Q. (2022). Machine learning based customer meta-combination brand equity analysis for marketing behavior evaluation. *Information Processing & Management*.

[23] Rajendran S., Khalaf O. I., Alotaibi Y., Alghamdi S. (2021). MapReduce-based big data classification model using feature subset selection and hyperparameter tuned deep belief network. *Scientific Reports*.

[24] Kumar A., Kabra G., Mussada E. K., Dash M. K., Rana P. S. (2019). Combined artificial bee colony algorithm and machine learning techniques for prediction of online consumer repurchase intention. *Neural Computing & Applications*.

[25] Shen Y., Wang Z., Shen Bo., Alsaadi F., Alsaadi F. E. (2020). Fusion estimation for multi-rate linear repetitive processes under weighted try-once-discard protocol. *Information Fusion*.

